The article "miR-517a is up-regulated in glioma and promotes glioma tumorigenesis in vitro and in vivo" was retracted in 2023. Reasons: manipulated images; duplicated images; signs of a paper mill.

# miR-517a is up-regulated in glioma and promotes glioma tumorigenesis *in vitro* and *in vivo*

**DOI:** 10.1042/BSR20181196

**Published:** 2019-05-02

**Authors:** Cheng-li Du, Fei Peng, Ke-qin Liu

**Affiliations:** Department of Neurosurgery, Nanxishan Hospital of Guangxi Zhuang Autonomous Region, Chongxin Road No. 46, Guilin 541002, Guangxi Zhuang Autonomous Region, China

**Keywords:** apoptosis, glioma, invasion, migration, miR-517a, proliferation

## Abstract

miR-517a has been reported to act as an oncogenic miRNA in human hepatocellular carcinoma and lung cancer. However, the roles and underlying molecular mechanism of miR-517a in glioma remain unclear. In the present study, the expression of miR-517a in clinical glioma tissues and glioma cell lines was examined by quantitative real-time PCR (qRT-PCR). Transfected with knockdown or forced expression of miR-517a, the effects of miR-517a on cell proliferation, migration, and invasion were detected through *in vitro* and *in vivo* tumorigenesis assays. Here, we report that miR-517a expression was up-regulated in glioma tissues when compared with normal brain tissues, and up-regulation of miR-517a level is tightly correlated with the status of pathology classification of glioma. A functional assay found that overexpression of miR-517a in glioma cells markedly promoted or suppressed cell proliferation, colony formation, migration and invasion, respectively. Moreover, we revealed that the knockdown of miR-517a dramatically suppressed glioma cell growth, migration, and invasion *in vitro* and *in vivo*. Furthermore, we found that knockdown of miR-517a significantly induced apoptosis. Therefore, miR–517a acts an oncogenic miRNA that promotes tumor progression in glioma, and thus may become a promising therapeutic candidate for glioma.

## Introduction

Malignant gliomas are the most common primary tumors of the central nervous system. They are characterized by high invasion, migration, and proliferation abilities [1–3]. Despite recent advances in our understanding of the molecular mechanisms of the disease – and improvement in therapeutic strategies – the median survival of GBM patients still remains dismal, with less than 1 year after diagnosis [4]. Thus, it is quite urgent to understand the molecular mechanisms by which glioma initiates, progresses, invades, and recurs in order to develop effective prognostic biomarkers and novel therapies.

miRNAs are endogenous, small, non-coding RNAs that regulate gene expression by antisense complementarity to specific mRNA. MiRNAs are short non-coding RNAs that interfere with target gene expression through either inhibition of mRNA translation or promotion of mRNA degradation [5]. Recent works have suggested that deregulation of a group of small non-coding RNAs called miRNAs is involved in initiation and progression of gliomas, including miR-335 [6], miR-218 [7], miR-15b, miR-152 [8], miR-92b [9], miR-145 [10], and miR-124 [11]. miR-517a is considered to be a novel oncomiR and was observed to be elevated in human hepatocellular carcinoma (HCC) [12]; expression of miR-517a increased proliferation, migration, and invasion of HCC cells *in vitro* [12]. A recent study reported that miR-517a accelerated lung cancer cell proliferation, migration, and invasion through inhibiting forkhead box J3 (FOXJ3) expression [13]. However, the regulatory mechanism of miR-517a in glioma remains largely unclear.

The article "miR-517a is up-regulated in glioma and promotes glioma tumorigenesis in vitro and in vivo" was retracted in 2023. Reasons: manipulated images; duplicated images; signs of a paper mill.

In the present study, we investigated the putative role of miR–517a in the progression of glioma. We found that the expression of miR–517a was frequently increased in clinical glioma tissue samples compared with normal brain tissues, and up-regulation of miR–517a level is tightly correlated with the status of pathology classification. Furthermore, through *in vitro* and in mouse xenograft model, we investigated the function of miR-517a in glioma, including the proliferation, migration, invasion, and apoptosis.

## Materials and methods

### Clinical samples

We obtained 60 snap-frozen glioma and 20 normal brain samples from Nanxishan Hospital of Guangxi Zhuang Autonomous Region, including 20 grade II tumors, 20 grade III tumors, and 20 grade IV tumors according to the WHO classification. All specimens had confirmed pathological diagnosis and were classified according to the WHO criteria (Table 1). These glioma cases were from 38 males and 22 females with age ranging from 19 to 72 years. The purpose and content of the present study were explained fully to all subjects, whose signed informed consent was obtained prior to enrollment. Written informed consent was obtained from each patient. Our study was conducted in accordance with the World Medical Association’s Helsinki guidelines and was approved by the Research Ethics Committee of Nanxishan Hospital of Guangxi Zhuang Autonomous Region, China.

**Table 1:** Clinicopathological data of the patients included in the present study

	Number of patients
**All patients**	60
**Gender**	
**Male**	38
**Female**	22
**Age**	
**<65 year old**	42
**≥65 year old**	18
**Grade**	
**I**	20
**II**	20
**III**	20

### Cell lines

The LN18, U87, and U118 glioma cell lines and primary normal human astrocytes (NHAs) were purchased from the Institute of Biochemistry and Cell Biology of the Chinese Academy of Sciences (Shanghai, China). Cells were cultured in DMEM (GIBCO-BRL) medium supplemented with 10% fetal bovine serum (FBS), 100 U/ml penicillin and 100 mg/ml streptomycin (Invitrogen, Carlsbad, CA, U.S.A.) at 37°C/5% CO_2_. All cell lines were authenticated by short tandem repeat DNA profiling.

The article "miR-517a is up-regulated in glioma and promotes glioma tumorigenesis in vitro and in vivo" was retracted in 2023. Reasons: manipulated images; duplicated images; signs of a paper mill.

### RNA isolation, reverse transcription, and qRT-PCR

Total RNA was isolated with Trizol reagent (Invitrogen) according to the manufacturer’s instructions. Total RNA (500 ng) was reverse transcribed in a final volume of 10 μl using random primers under standard conditions for the PrimeScript RT reagent Kit (TaKaRa, Dalian, China). We used the SYBR Premix Ex Taq (TaKaRa, Dalian, China) to determine ANRIL expression levels, following the manufacturer’s instructions. For miR-517a, RNA was transcribed into complementary DNA and amplified with specific sense, 5′ -ATTGGGGCTCGCGT-3′, according to the manufacturer’s instructions (Takara Bio, Inc.). U6 (sense primer: 5′-CTCGCTTCGG CAGCACATATA-3′) genes were used as miRNA and gene internal controls, respectively. Cycling conditions were 95°C for 10 min to activate DNA polymerase, followed by 45 cycles of 95 °C for 15 s, 58 °C for 15 s, and 72 °C for 10 s. Specificity of amplification products was confirmed by melting curve analysis. PCR reactions for each gene were repeated three times. Independent experiments were done in triplicate.

### Stable expression or knockdown of miR-517a in glioma cell lines

Lentiviral vectors which overexpressed or knockdown miR-517a were purchased from GenePharma (Shanghai, China). A lentiviral vector expressing scrambled RNA was used as the control and the sequence was 5′-TTAACGTCGATGTCCGT-3′. Glioma cell lines were infected with lentiviral vector. Total RNA from these cell clones was isolated, and levels of miR-517a were quantified using RT-qPCR.

### Western blot assay and antibodies

Cells were lysed using mammalian protein extraction reagent RIPA (Beyotime) supplemented with protease inhibitors cocktail (Roche) and phenylmethylsulfonyl-fluoride (Roche). Fifty micrograms of protein extractions were separated by 10% SDS–PAGE, transferred to 0.22 mm nitrocellulose (NC) membranes (Sigma) and incubated with specific antibodies. Autoradiograms were quantified by densitometry (Quantity One software; Bio-Rad). Information on the antibodies is provided: Bad (1:1000 dilution CST- 9292); Bax (1:1000 dilution CST- 2772); Bcl-2 (1:1000 dilution CST- 15071); Cleaved Caspase-3 (1:1000 dilution CST- 9661), and β-actin (1:1000 dilution CST-4970).

### MTT assay

A cell proliferation assay was conducted with MTT kit according to the manufacturer’s instruction. Triplicate wells were measured in each treatment group.

### Colony formation assay

For the cells to form colonies, a total of 600 LN18 or U118 cells transfected with miR–517a mimic or scramble mi-RNA were placed onto a fresh six-well plate and maintained in media containing 10% FBS, replacing the medium every 4 days. After 2 weeks, the colonies were fixed with methanol and stained with 0.1 % crystal violet (Sigma, St. Louis, MO). The visible colonies were manually counted. Triplicate wells were assessed for each treatment group.

The article "miR-517a is up-regulated in glioma and promotes glioma tumorigenesis in vitro and in vivo" was retracted in 2023. Reasons: manipulated images; duplicated images; signs of a paper mill.

### Transwell assay

Matrigel-coated invasion chambers (8 μm, BD Biosciences, San Jose, CA, U.S.A.) were prepared according the manufacturer’s instructions. Transfected GBM cells were seeded in the upper compartment and allowed to migrate for 24 h in an incubator. Cells were seeded in 1% FBS DMEM medium in the upper chamber and 10% FBS medium in the well below the insert. The cells that had invaded the lower surface were fixed with 4% paraformaldehyde and stained with 0.1% crystal violet. The number of cells that had invaded through the Matrigel was counted in six random fields for triplicate membranes under the microscope.

### Flow-cytometric analysis

After the double staining with FITC-Annexin V and propidium iodide (PI) was done using the FITC Annexin V Apoptosis Detection Kit (BD Biosciences) according to the manufacturer’s recommendations, the cells were analyzed with a flow cytometry (FACScan®; BD Biosciences) equipped with a CellQuest software (BD Biosciences). Cells were discriminated into viable cells, dead cells, early apoptotic cells and apoptotic cells, and then the relative ratio of early apoptotic cells were compared with control transfectant from each experiment. Cells for cell cycle analysis were stained with PI using the CycleTEST™ PLUS DNA Reagent Kit (BD Biosciences) following the protocol and analyzed by FACScan.

## Tumor formation assay in a nude mouse model

Female athymic BALB/c nude mice (4-week-old) were maintained under pathogen-free conditions and manipulated according to protocols approved by the Shanghai Medical Experimental Animal Care Commission. U87 cells were stably transfected with sh-miR-517a and empty vector and harvested from 6-well cell culture plates. A total of 100 μl of suspended cells was subcutaneously injected into a single side of the posterior flank of each mouse. Tumor growth was examined every 3 days, and tumor volumes were calculated using the equation V = 0.5 × D × d2 (V, volume; D, longitudinal diameter; d, latitudinal diameter). At 18 days post-injection, mice were killed, and the subcutaneous growth of each tumor was examined.

### Statistical analysis

The Student’s *t* test (two-tailed), one-way ANOVA, and Mann–Whitney *U* test were conducted to analyze the *in vitro* and *in vivo* data by SPSS 20.0 software. *P*-values less than 0.05 were considered significant.

The article "miR-517a is up-regulated in glioma and promotes glioma tumorigenesis in vitro and in vivo" was retracted in 2023. Reasons: manipulated images; duplicated images; signs of a paper mill.

## Results

### Up-regulation of miR-517a in human glioma tissues and cell lines

To explore the expression and significance of miR-517a in glioma, we first examined the expression level of miR-517a in 60 snap-frozen glioma tissues and 20 normal brain tissues by quantitative real-time PCR (qRT-PCR). Compared with normal brain tissues, significant increase of miR-517a was observed in glioma tissues (Figure 1A). Meanwhile, we also observed that increased levels of miR-517a in glioma patients were positively correlated with the status of pathology classification (WHO II vs WHO IV; *P*<0.01). A gradually increased miR-517a expression was found from grade II to IV samples (Figure 1A). In addition, qRT-PCR was performed on a panel of three human glioma cell lines (LN18, U87, and U118) and primary NHA. Up-regulation of miR-517a could also be observed in glioma cell lines than that of NHA (Figure 1B). These results suggested that miR-517a could be closely related to human glioma and up-regulation of miR-517a might be related to glioma oncogenesis and progression.

**Figure 1:** miR-517a expression is up-regulated in glioma tissue samples and cell lines (**A**) The expression levels of miR-517a in glioma tissues and normal brain tissues were determined by qRT-PCR. U6 was used as a loading control. Increased levels of miR-517a was positively correlated with the status of pathology classification by qRT-PCR. The unpaired *t*test was used for this assay. (**B**) Expression levels of miR-517a in three glioma cell lines (LN18, U87, and U118) and primary NHAs were determined by qRT-PCR. *P<0.05 and **P<0.01 vs NHAs.

### Overexpression of miR-517a promotes growth of glioma cells *in vitro*

To further explore its biological roles in glioma, miR-517a overexpression lentiviral vector (Lv-miR-517a) and lentiviral empty vector (miR-NC) were transfected into human glioma LN18 and U118 cells. After transfection, the expression level of miR-517a was significantly up-regulated compared with the control group (Figure 2A). We then performed colony formation assay to determine the cell proliferation in each group, and showed that up-regulation of miR-517a significantly increased LN18 and U118 cells proliferation (Figure 2B,C). Additionally, MTT assay indicated that up-regulation of miR-517a also substantially promoted the proliferation ability in LN18 and U251 cells (Figure 2D). These results demonstrated that miR-517a could promote the proliferation phenotype of glioma cells *in vitro*.

**Figure 2:** miR-517a promotes glioma cell growth *in vitro* (**A**) Real-time RT-PCR was conducted to determine the relative miR–517a level in glioma LN18 and U118 cells transfected with miR–517a mimic or scramble miR-NC. (**B,C**) *In vitro* proliferative ability of glioma cells was significantly decreased in overexpressed miR-517a cells compared with miR-NC cells by colony formation assay in LN18 (upper) and U118 (lower) cells. (**D**) MTT assay was performed to determine cell proliferation in LN18 (upper) and U118 (lower) cells. Non-transfected LN18 and U118 cells were used as control. Absorbance was read at 490 nm with averages from triplicate wells. Data are presented as mean ± SD from three independent experiments. **P<0.01 and ***P<0.005 vs miR-NC.

The article "miR-517a is up-regulated in glioma and promotes glioma tumorigenesis in vitro and in vivo" was retracted in 2023. Reasons: manipulated images; duplicated images; signs of a paper mill.

### Overexpression of miR-517a induced the invasion and migration of glioma cells *in vitro*

Next, we examined the effects of miR-517a on the ability of LN18 and U118 cells to invade and migrate. Cell migration and invasion abilities were determined in the LN18 and U251 cells transfected with the Lv-miR-517a or miR-NC by a transwell chamber or a Boyden chamber, respectively. Transwell assays with Matrigel demonstrated that LN18 and U118 cells-overexpressing miR-517a were found to have significantly increased migration and invasion abilities than control cells (Figure 3). Together, these data suggest that miR-517a is critical for glioma cells invasion and migration *in vitro*.

**Figure 3:** miR-517a promotes migration and invasion of glioma cells *in vitro* (**A**) Representative images of transwell invasion assay using LN18 and U118 cells stably expressing miR-517a or mi-NC. (**B**) Stably up-regulating miR-517a increased the migration and invasiveness ability of LN18 and U118 cells *in vitro.* Data are presented as mean ± SD from three independent experiments. **P<0.01 and ***P<0.005 vs miR-NC.

### Knockdown of miR-517a inhibits glioma cell proliferation, migration, and invasion

To determine whether miR-517a had an effect on the malignant phenotype of glioma cells, we constructed lentiviral-mediated knockdown of miR-517a in the U87 cell line, which exhibited the highest miR-517a expression level among cell lines in our study. The miR-517a expression levels were knocked down more than 70% in U87 cell line relative to the control group (Figure 4A). Colony formation assay and MTT assay showed that knockdown of miR-517a decreased the proliferation ability in U87 cells (Figure 4B,C). In addition, the transwell assays demonstrated that LN18 cells knockdown of miR-517a were found to have significantly reduced the migration and invasion abilities than control cells (Figure 4D).

**Figure 4:** Effects of knockdown of miR-517a on the growth, migration, and invasion of glioma cells *in vitro* (**A**) U87 cells were transduced with anti-miR-517a or control. (**B**) Colony-forming assays were conducted to determine the proliferation of anti-miR-517a-transfected U87 cells. (**C**) MTT assays were used to determine the cell viability of anti-miR-517a-transfected U87 cells. Values represented the mean ± SD from three independent experiments. (**D**) Representative images of transwell invasion assay using U87 cells transduced with anti-miR-517a or mi-NC. (B) Knockdown of miR-517a decreased the migration and invasiveness ability of U87 cells *in vitro*. Data are presented as mean ± SD from three independent experiments. **P<0.01 and ***P<0.005 vs miR-NC.

The article "miR-517a is up-regulated in glioma and promotes glioma tumorigenesis in vitro and in vivo" was retracted in 2023. Reasons: manipulated images; duplicated images; signs of a paper mill.

### Knockdown of miR-517a induces apoptosis *in vitro*

To illustrate the mechanisms of how miR-517a modulates glioma cell growth, flow cytometry was applied to detect the effects of miR-517a on cell apoptosis. Annexin V/PI double staining demonstrated that the proportion of apoptosis LN18 cells transfected with anti-miR-184 was significantly higher than that in the anti-miR-NC group (Figure 5A). Concordantly, the expression of caspase-3 cleavage and Bad were activated, the expression of Bax and Bcl-2 were markedly reduced in LN18 cells transfected with anti-miR-517a (Figure 5B).

**Figure 5:** miR-517a knockdown induces apoptosis in U87 cell (**A**) Apoptosis in U87 cell transduced with anti-miR-517a and control was performed by flow cytometry and the apoptotic index was defined as the percentage of apoptotic cells. **P<0.01. (**B**) Cleaved caspase-3, Bax, Bad2, and Bcl-2 were evaluated by Western blotting. The data represent the mean ± SD from three independent experiments. **P<0.01 vs miR-NC.

### Down-regulation of miR-517a inhibits glioma cell tumorigenesis *in vivo*

To explore whether the level of miR-517a expression could affect tumorigenesis, LN18 cells stably transfected with lentiviral-mediated anti-miR-517a or empty vector were inoculated into female nude mice. Eighteen days after the injection, the tumors formed in the anti-miR-517a group were substantially smaller than those in the control group (Figure 6A,B). Moreover, the mean tumor weight at the end of the experiment was markedly lower in the anti-miR-517a group compared with the empty vector group (Figure 6C). Tumors formed from lentiviral anti-miR-517a-transfected LN18 cells exhibited decreased positivity for Ki67 than those from control cells (Figure 6D). These findings indicate that knockdown of miR-517a inhibits tumor growth *in vivo*.

**Figure 6:** Effects of down-regulation of miR-517a on tumor growth *in vivo* (**A**) The tumor volume was calculated once every 3 days after injection of U87 cells stably transfected with sh-miR-517a or empty vector. Points, mean (*n*=7); bars indicate SD. (**B**) Tumor weights are represented as means of tumor weights ± SD. (**C**) Tumor growth curves are summarized. The error bars indicate the SD. (**D**) Tumors developed from sh-miR-517a-transfected U87 cells showed lower Ki67 protein levels than tumors developed by control cells. Upper: H&E staining; Lower: immunostaining. *P<0.05, **P<0.01, and N.S. not significant.

The article "miR-517a is up-regulated in glioma and promotes glioma tumorigenesis in vitro and in vivo" was retracted in 2023. Reasons: manipulated images; duplicated images; signs of a paper mill.

## Discussion

Gliomas are well-known for not only rapid proliferation but also invading the surrounding brain tissue, leading to extremely poor prognosis. Similar to other tumors, some environmental carcinogenic factors may also be associated with the occurrence of glioma [14]. miRNAs have emerged as key factors involved in several biological processes, including development, differentiation, cell proliferation, and tumorigenesis [15,16]. Thus, it is possible that miRNAs may shed light on the potential mechanism of glioma. In the present study, our data provided the first evidences that expression of miR-517a was increased in glioma tissues compared with normal brain tissues. We further found that miR-517a expression was positively correlated with the status of pathology classification. These results suggest that miR-517a may promote the progression of glioma.

Chromosome 19 miRNA cluster (C19MC) on 19q13.41 have been considered so far to be the largest human miRNA gene cluster, which harbor 43 miRNA genes and extends over 100 kb long region [17]. Recent miRNA-related studies show that miR–517a has been proposed to be promoted in tumor metastasis of HCC and lung cancer [12,13]. Whereas, in bladder cancer miR-517a was down-regulated, and ectopic restoration of miR-517a significantly inhibited cell proliferation by promoting apoptosis [18]. These studies suggest that miR–517a may have have different roles in different cancers. To comprehensively understand the effect of miR-517a on glioma cancer cells, we performed *in vitro* proliferation and invasion assays to identify the migration and invasion ability of glioma cells. Importantly, our study showed that knockdown of miR–517a significantly inhibited tumorigenesis as well as the tumor growth of glioma cells *in vivo*. These data further indicate that miR-517a indeed acts as a novel oncogenic miRNA in glioma cells.

Apoptosis, a fundamental process essential for development and maintenance of tissue homeostasis, is a major mechanism to eliminate cancer cells [19]. Thus, an effective strategy for cancer treatment seems to target signaling intermediates in the apoptosis-inducing pathways [20]. Here, we showed that knockdown of miR-517a induces apoptosis in LN18 cells. Consistently, the expression of caspase-3 cleavage and Bad were up-regulated, the expression of Bax and Bcl-2 were markedly down-regulated in LN18 cells transfected with anti-miR-517a, which is consistent with apoptosis induction. These data add further evidence for the oncogenesis role of miR-517a in glioma.

The article "miR-517a is up-regulated in glioma and promotes glioma tumorigenesis in vitro and in vivo" was retracted in 2023. Reasons: manipulated images; duplicated images; signs of a paper mill.

In summary, our results showed that miR-517a expression was frequently up-regulated in glioma specimens and cell lines, and increased levels of of miR–517a level was tightly correlated with the malignant progression. Our study *in vitro* and *in vivo* suggested that miR–517a acts as a novel oncogenic miRNA that promotes tumor cell proliferation, migration, and invasion of glioma cells by inducing apoptosis. The present study provides novel insights into the mechanism underlying the development and progression of glioma, and suggests that miR–517a may become a promising therapeutic candidate for glioma.

## Abbreviations

Bad: Bcl-2-associated death promoter
Bax: Bcl-2-associated X protein
Bcl-2: B-cell lymphoma-2
FBS: fetal bovine serum
GBM: glioblastoma multiforme
HCC: hepatocellular carcinoma
MTT: Methylthiazolyldiphenyl-tetrazolium bromide
NHA: normal human astrocyte
PI: propidium iodide
qRT-PCR: quantitative real-time PCR
RIPA: Radio-Immunoprecipitation Assay
